The article "A Validated RP-HPLC Method for Simultaneous Determination of Cefixime and Clavulanic Acid Powder in Pediatric Oral Suspension" was published in 2022. Journal: Int J Anal Chem.

# A Validated RP-HPLC Method for Simultaneous Determination of Cefixime and Clavulanic Acid Powder in Pediatric Oral Suspension

**DOI:** 10.1155/2022/8331762

**Published:** 2022-07-01

**Authors:** Utsav Nepal, Vijay Kumar Panthi, Namindra Prasad Chaudhary, Samip Chaudhary

**Affiliations:** ^1^Department of Pharmacy, Kathmandu University, School of Science, Dhulikhel, Nepal; ^2^Quality Control Department, Royal Sasa Nepal Pharmaceuticals, Bharatpur-18 44200, Chitwan, Nepal; ^3^Research and Development Department, Royal Sasa Nepal Pharmaceuticals, Bharatpur-18 44200, Chitwan, Nepal; ^4^Department of Pharmacy, Tribhuvan University, Sunsari Technical College, Sunsari, Nepal; ^5^Research and Development Department, Asian Pharmaceuticals, Rupandehi, Nepal; ^6^Research and Development Department, Corel Pharmaceuticals, Rupandehi, Nepal; ^7^Kantipur College of Medical Science, Tribhuvan University, Sitapaila, Kathmandu, Nepal; ^8^Tri-Chandra Multiple Campus, Tribhuvan University, Kathmandu, Nepal

## Abstract

A new reverse phase high-performance liquid chromatography (RP-HPLC) method was developed and validated for the simultaneous estimation of pediatric oral powder formulation containing cefixime (CFX) and clavulanic acid (CVA). In this research, an analytical C18 (4.6 mm × 25 cm), 5 *μ*m column was used for chromatographic separation with a mixture of methanol and water containing disodium hydrogen phosphate in ratio of 20 : 80 v/v as the mobile phase (pH 5.5 adjusted with orthophosphoric acid) at a flow rate of 1.0 mL/min. The detecting wavelength and run time were 220 nm and 15 min, respectively. Moreover, the column temperature was maintained at 30°C. The analytical method was validated prior to meeting the conditions specified by International Conference on Harmonization (ICH) and the parameters were specificity, linearity, limit of detection (LOD), limit of quantification (LOQ), accuracy, precision, robustness, and solution stability. The calibration curve was found to be linear between the concentration ranges of 0.024–0.036 mg/mL and 0.032–0.048 mg/mL for CFX and CVA, respectively. Furthermore, the LOD and LOQ of CFX were 0.0008 and 0.0025 *μ*g/mL, respectively. Accordingly, LOD and LOQ of CVA were 0.0021 and 0.0065 *μ*g/mL, respectively. The accuracy of the optimized method was examined by recovery studies and the mean recovery was observed to be 98.96% and 99.05% for CFX and CVA, respectively, at 100% spiked level. The repeatability testing for both standard and sample solutions revealed that the method is precise within the acceptable range and the %RSD of the precision was <2%. In addition, the findings of specificity, linearity, accuracy, precision, robustness, LOD, LOQ, and solution stability studies of both CFX and CVA were within the criteria of acceptable limit as well.

The article "A Validated RP-HPLC Method for Simultaneous Determination of Cefixime and Clavulanic Acid Powder in Pediatric Oral Suspension" was published in 2022. Journal: Int J Anal Chem.

## 1. Introduction

Cephalosporins are antimicrobial agents that belong to the beta-lactam class which are broadly used to treat several infections caused by Gram-positive and Gram-negative bacteria. Cephalosporins are categorized into five generations according to their range of spectrum against these bacteria [1]. The third-generation cephalosporins are widely applied for the treatment of several types of infections in children. Currently, cefixime (CFX) is the only third-generation cephalosporin for oral delivery in Canada, and the license was approved in 1990. The gastrointestinal absorption of CFX is incomplete, approximately 40–50% is absorbed, and the oral suspension is completely absorbed in a rapid manner in comparison with tablets [2]. The recommended oral dosage for children is 8 mg/kg once a day or in two divided doses. Various studies have revealed that CFX has better activity against streptococci (group A and group B) and *Streptococcus pneumonia.* However, viridans streptococci and groups C, F, and G streptococci are only considered as a moderately vulnerable, whereas *Staphylococcus aureus*, coagulase-negative staphylococci, enterococci, and *Listeria monocytogenes* are resistant [3]. Till date, no abundant published study has exhibited efficacy for the cure of children suffering from sinusitis, bronchitis, or pneumonia. However, the antimicrobial spectrum of CFX does entail the bacterial pathogens that generally cause sinusitis and pneumonia in children. Moreover, CFX is highly effective for the management of young children having gastroenteritis caused by *Salmonella* and *Shigella* species that are resistant to conventional antibiotics including amoxicillin and trimethoprim-sulfamethoxazole. However, the possibility of CFX resistance development against these pathogens is still unknown with the enhanced use in upcoming days [4, 5].

On the other hand, potassium clavulanate (PCV) is a potassium salt having clavulanate as the counterion. It acts as a suicide inhibitor of bacterial beta-lactamase enzymes and has only weak antibiotic activity when administered alone. However, it can be used in combination with amoxicillin trihydrate for treatment of several bacterial infections, where it avoids antibiotic inactivation by microbial lactamases [6, 7]. Moreover, PCV is a vital beta-lactam antibiotic that increases the antibacterial action of both penicillin and cephalosporin over various resistant strains of bacteria. Enhancing resistance to cephalosporins, in these days, the combinational delivery of cephalosporins and beta-lactamase inhibitor such as clavulanic acid (CVA) is becoming more prevalent in order to increase the antibacterial action of cephalosporins [8]. Furthermore, CVA is a drug of first choice for infections associated with skin, soft tissue, and urinary tract and for surgical prophylaxis. The oral absorption of CVA is good and absorption is not impacted by ingesta. It permeates insufficiently into milk and CSF and across the blood-prostate and blood-bronchus barriers (regardless of the degree of inflammation) in an insignificant manner. Excretion is mainly by glomerular filtration, producing high clavulanate concentrations in urine. Formulations for use in dogs and cats provide 1.25 mg of CVA for each 5 mg of amoxicillin and the half-life of PCV is shorter as compared to amoxicillin due to extensive metabolism [9].

The article "A Validated RP-HPLC Method for Simultaneous Determination of Cefixime and Clavulanic Acid Powder in Pediatric Oral Suspension" was published in 2022. Journal: Int J Anal Chem.

In the case of analytical methods, there are various literature that have been suggested for separate analysis of CFX and CVA. Recently, antibiotic susceptibility testing of isolates was also carried out using a standard disk diffusion test and the VITEK 2 compact system, using a Gram-negative antibiotic susceptibility card [10]. However, until these days, it has been very difficult to find appropriate studies that aid in the simultaneous determination of these two drugs. Several analytical methods have been recommended for the analysis of CFX and other antibiotics after complexation and derivatization with a variety of chemical reagents. These approaches include capillary electrophoresis, voltammetric method, spectrophotometric methods, HPLC/tandem mass spectrometry, and IPLC (ion-pairing liquid chromatography). Moreover, among these methods, UV/Vis spectrophotometry is considered one of the most widely used techniques for evaluation of CFX after derivatization [11–13]. Furthermore, sufficient studies are also available for simultaneous estimation of CVA and amoxicillin trihydrate and CVA and ticarcillin in bulk and pharmaceutical formulations using UV spectrophotometry, HPLC, and so forth. In addition, a validated HPLC method is also suggested for assessment of CFX and PCV in tablet dosage form at the same time [14, 15]. However, till date, no suitable analytical methods for simultaneous determination of CFX and CVA in pediatric oral powder have been available. Furthermore, the analytical method validation by HPLC is a vital task which ensures that techniques shall provide authenticated and repeatable results; it is a pivotal step in development of new dosage forms as it provides information about several validation parameters such as accuracy, linearity, precision, and detection and quantitation limits. Currently, submitting validation data to the regulatory authorities is mandatory for pharmaceutical companies. Additionally, requirements associated with analytical method validations were accommodated and accessible from different institutions including ICH (International Conference on Harmonization) and FDA [16, 17]. Therefore, the main objective of this research is to develop and validate appropriate analytical methods by HPLC for analysis of these drugs simultaneously in pediatric oral powder formulation.

The article "A Validated RP-HPLC Method for Simultaneous Determination of Cefixime and Clavulanic Acid Powder in Pediatric Oral Suspension" was published in 2022. Journal: Int J Anal Chem.

## 2. Materials and Methods

### 2.1. Chemicals and Reagents

A formulated sample of oral powder containing cefixime and clavulanic acid was obtained from the research and development department of our company. Methanol (HPLC grade), water (HPLC grade), disodium hydrogen phosphate, and potassium dihydrogen phosphate (analytical reagent grade) were purchased from Thermo Fisher Scientific India Ltd.

### 2.2. Instrumentation

The below-mentioned instruments were applied for the evaluation of formulated oral powder. Agilent 1260 (infinity II) HPLC system was utilized for the development and validation of liquid chromatography (Waldron, Germany), facilitated with a pump (model: G7116A), an autosampler (ALS) (model: G7129A), and a C18 (250 cm × 4.6 mm), 5 *μ*m column (Paisley, UK), and the detector included UV/VIS operated at 220 nm. Agilent OpenLab Software (version 3.2.0.0) was used in order to process and evaluate the obtained results. Additionally, analytical balance demonstrating four digits was used (Radwag, model: AS 220.X2, Poland) for weighing purpose and sonicator (MRC, model: ACP-150H, India) was used prior to dissolving the reagents.

### 2.3. Chromatographic Conditions

The diluent was prepared by dissolving 7.10 g of disodium hydrogen phosphate in 500 mL water and pH was adjusted to 7.0 with potassium dihydrogen phosphate solution. Furthermore, the mobile phase was prepared by dissolving 3.408 g of disodium hydrogen phosphate in 800 mL water (HPLC grade) and then 200 mL methanol was added and finally pH was adjusted to 5.5 with orthophosphoric acid. The mobile phase was filtered through 0.45 *μ*m membrane filters and degassing was done by sonication for 20 min. The analysis was performed on an Agilent 1260 HPLC system. The analyses were carried out on an analytical column C18, 5 *μ*m, 250 × 4.6 mm with detection wavelength of 220 nm by a UV/VIS detector. Moreover, the operating temperature of the column was set to 30°C. The injection volume and flow rate were 20 *μ*L and 1.0 mL/min, respectively, in addition to runtime of 15 minutes.

### 2.4. Preparation of Standard Solution

Accurately weighed about 30 mg reference standard (RS) of cefixime trihydrate and 40 mg RS of CVA was then transferred to a 50 mL volumetric flask. Subsequently, 40 mL of diluent was added into it and sonicated for 20 minutes. The volume was made up of diluent, shaken well, and filtered. Additionally, 5 mL of this solution was further diluted with 100 mL of diluent; shaking was done properly and filtered. The final concentration was 0.030 mg/mL and 0.04 mg/mL of CFX and CVA, respectively.

The article "A Validated RP-HPLC Method for Simultaneous Determination of Cefixime and Clavulanic Acid Powder in Pediatric Oral Suspension" was published in 2022. Journal: Int J Anal Chem.

### 2.5. Preparation of Sample Solution

Approximately 11 g of sample powder (dry syrup) was weighed and transferred to a clean and dry 30 mL HDPE bottle. The distilled water was added up to the mark on the bottle and shaken vigorously. In addition, it weighed accurately as near as 2.7 g of the reconstituted suspension in a 50 mL beaker. 20 mL of diluent was added further and stirred with the aid of a glass rod for a few minutes and carefully transferred to a 50 mL volumetric flask with the help of a funnel. The final volume was adjusted with diluents with proper shaking and filtered. Finally, pipette out 5 mL of this solution and further dilute it to 95 mL with diluent.

### 2.6. Method Validation

#### 2.6.1. Specificity

Specificity is considered the vital part of HPLC which deals with the potentiality of analytical techniques to differentiate between the analyte and other ingredients in the composite mixture [17]. In this study, in order to examine the specificity of the approached method, 20 *μ*L of one blank solution, one placebo solution, standard solution of CFX and CVA (5 measurements each), and sample solution of CFX and CVA (5 measurements each) was separately injected at 100% concentration. The retention times of CFX and CVA in standard solution and sample solution were identified and compared.

#### 2.6.2. Linearity and Range

Linearity is defined as the ability to find the test values which have direct relationship to the concentration of the analyte. In this study, linearity was evaluated by injecting three replicates of five different concentrations of CFX (0.024, 0.027, 0.03, 0.033, and 0.036 *μ*g/mL) and CVA (0.032, 0.036, 0.04, 0.044, and 0.048 *μ*g/mL). The mean peak areas of CFX and CVA were plotted against concentrations. Subsequently, the linearity was examined with the help of calibration curve to assess coefficients of correlation, slope, and intercept. Generally, a value of correlation coefficient (*r*^2^) > 0.998 is considered the evidence of an acceptable fit for the data to the regression line [18].

#### 2.6.3. Accuracy

In this study, assay method of this parameter was examined by recovery analysis at different concentration levels including 80%, 100%, and 120%. The three replicates of each concentration of both CFX and CVA were injected. The recovery percentage of both CFX and CVA added and finally RSD were determined for each of the analyzed samples.

The article "A Validated RP-HPLC Method for Simultaneous Determination of Cefixime and Clavulanic Acid Powder in Pediatric Oral Suspension" was published in 2022. Journal: Int J Anal Chem.

#### 2.6.4. Precision

Precision deals with the degree of closeness among individual tests, when repetitive technique was applied in order to evaluate multiple replicates in three different occasions [19]. In this study, the system precision and method precision (repeatability) of the proposed methods were determined by several measurements of standard and sample solution, respectively. The system precision was assessed by six measurements of the standard solution at the 100% concentration levels on the same day. Moreover, method precision was examined by six assay measurements of the sample solution at the 100% concentration levels on the same day. The %RSD of the observed values was assessed prior to examining the repeatability results.

#### 2.6.5. Limit of Detection (LOD) and Limit of Quantitation (LOQ)

The limit of detection (LOD) is defined as lesser quantity of analyte in a sample which can be estimated but not inevitably assessed. Similarly, the limit of quantification (LOQ) deals with the minimum portion of analyte in a sample that can be quantifiably evaluated with appropriate precision [20]. The calibration curve was repeatedly used for 6 times and SD of the intercepts was evaluated using the below-mentioned formula to calculate the values of LOD and LOQ.

(1) $$\begin{array}{c} \text{LOD}=\frac{\left(3{\text{.}3}^{*}\text{SD}\right)}{\text{Slope}}, \end{array}$$

(2) $$\begin{array}{c} \text{LOQ}=\frac{\left(10^{*}\text{SD}\right)}{\text{Slope}}, \end{array}$$

where SD is the standard deviation of *Y*-intercept of 6 calibration curves and Slope is the average slope of the 6 calibration curves [21, 22].

#### 2.6.6. Robustness

According to the International Conference on Harmonization (ICH), the robustness of an analytical procedure is defined by its ability to remain unaffected by small and deliberate variations in method parameters [23]. This parameter was assessed by studying the impact of minor variations in the chromatographic conditions. The conditions evaluated were different flow rates and pH of mobile phase. The flow rates and pH were altered by ±0.4 mL/min and ±0.4, respectively. The assay and %RSD of each sample were analyzed.

#### 2.6.7. Stability of Analytical Solutions

The stability of both analytical solutions (CFX and CVA) was assessed by determining the standard and sample preparations at 0 h and 24 h in the refrigerator and at ambient temperature of 30°C. Three injections from each solution were examined, and the average of the peak and the RSD were calculated.

## 3. Results and Discussion

### 3.1. Method Development and Optimization

The various physicochemical characteristics of both CFX and CVA were acquired from the previously published literature. The suitable analytical method was developed prior to selecting preliminary reverse phase HPLC-UV chromatographic conditions, such as stationary phase, mobile phase, determining wavelength, and procedure of sample preparation. Furthermore, in order to accomplish the goal, few attempts were done by varying the pH of mobile phase and optimizing the conditions of chromatographic separation on the C18 (250 × 4.6 mm), 5 *μ*m column. The result of method optimization is given in Table 1. Briefly, several pharmacopoeias have suggested the pH between 4.0 and 6.5 to be appropriate for the elution of cephalosporin related drugs and CVA. Therefore, we started from higher pH of 6.5 and gradually decreased it at the rate of 0.5. In the first trial, the pH of mobile phase was 6.5 and the resolution of peak was very poor; thereby we rejected this trial. Furthermore, in the second attempt, we decreased the pH to 6.0 prior to achieving better resolution but again we suffered the same problem. Thus, this attempt was also discontinued to apply further. Moreover, in the third trial, pH was decreased to 5.5 and finally obtained the good resolution in HPLC peak; therefore this method is optimized. However, to further examine the impact of lower pH, we decided to carry out few more trials. In the fourth, fifth, and sixth trial, the applied pH values were 5.0, 4.5, and 4.0, respectively, but in these trials we observed poor and unstable peak shape for both analytes. Thus, these trials including trial 1 and 2 are rejected and finally mobile phase having pH 5.5 (trial 3) was optimized and selected for detailed analysis of pediatric oral suspension containing CFX and CVA.

The article "A Validated RP-HPLC Method for Simultaneous Determination of Cefixime and Clavulanic Acid Powder in Pediatric Oral Suspension" was published in 2022. Journal: Int J Anal Chem.

The mobile phase contained 3.408 g disodium hydrogen phosphate dissolved in 800 mL water (HPLC grade) and 200 mL methanol in the ratio of 80 : 20 v/v and the pH was adjusted to 5.5 with orthophosphoric acid. The flow rate, injection volume, and the runtime were 1 mL/min, 20 *μ*L, and 15 min, respectively. Moreover, the operating column temperature was 30°C at wavelength of 220 nm using UV detector which was finalized as the appropriate chromatographic condition for the detailed study of this research, where both CFX and CVA were appropriately eluted revealing peak shape in a very symmetrical manner, resolution, and proper testing duration including retention time of approximately 7 min and 3 min for CFX and CVA, respectively.

### 3.2. Specificity

To determine specificity, 20 *μ*L solution from blank solution, placebo solution, standard solution of CFX and CVA (5 measurements each), and sample solution of CFX and CVA (5 measurements each) were separately injected at 100% concentration and the obtained chromatograms are shown in Figures 1–4. In this parameter, the result has been exhibited that there was not any asymmetrical HPLC peaks while analyzing the retention time of standard and sample solution of both CFX and CVA. In addition, the retention time of the major peak of both standard and sample solutions of CFX and CVA was compiled (Tables 2 and 3). Therefore, this result demonstrates that the peaks of analytes were pure as no peak interference was observed and these findings finally endorsed the specificity of the method.

### 3.3. Linearity and Range

Linearity in terms of analytical method deals with the capability of the method to achieve test results that are proportionally dependent on the concentration, over a specific range. The average peak area received from the HPLC analysis was represented with respect to different concentrations of each of CFX and CVA in order to get the calibration curve. In this study, the results of the linearity demonstrated a linear relationship over the concentration ranges of 0.024–0.036 mg/mL and 0.032–0.048 mg/mL for CFX (Figure 5) and CVA (Figure 6), respectively. Furthermore, the obtained correlation coefficient (*R*^2^) and regression equation of CFX were 0.997 and *y* = 38501*x* + 8.506, respectively. Similarly, in case of CVA, *y* = 15699*x* + 22.55 and *R*^2^ was found to be 0.992, demonstrating a linear interrelation between the analytes concentration and peak area.

### 3.4. Determination of LOD and LOQ

These parameters were assessed by determining LOD and LOQ as per the formula illustrated in Section 2.6.5. In this study, the LOD and LOQ of CFX were observed to be 0.0008 and 0.0025 *μ*g/mL, respectively. Accordingly, LOD and LOQ of CVA were 0.0021 and 0.0065 *μ*g/mL, respectively.

### 3.5. Accuracy

The accuracy of an analytical procedure deals with the vicinity of findings provided by the applied method in comparison with true value [20]. In this research, the results of accuracy revealed percentage recovery of CFX at all three levels (80%, 100%, and 120%) in the range of 98.24%–101.66% and %RSD values were in the range of 0.061–0.130% as given in Table 4. Similarly, percentage recovery of CVA at all three levels (80%, 100%, and 120%) was in the range of 98.16%–101.12% and %RSD values were in the range of 0.139–0.244% as given in Table 5. In this parameter, the percentage recovery at 80% and 100% concentration was within 98.0%–100%, while at 120% concentration level the percentage recovery was within 100.0%–102.0% which might be attributed to analyst error rather than systematic error as our linearity study exhibited the percentage recovery of all concentration levels (80%, 90%, 100%, 110%, and 120%) within 98.0%–100% (data not shown). In addition, similar results were obtained in a study done by Savadkouhi et al., where the percentage recovery was decreased gradually with increasing level of concentration [24]. In our accuracy study, the data of percentage recovery and %RSD were within the desired limits from 98.0% to 102.0% and not more than (NMT) 2.0%, respectively, which shows the usefulness of the method for routine drug analysis.

The article "A Validated RP-HPLC Method for Simultaneous Determination of Cefixime and Clavulanic Acid Powder in Pediatric Oral Suspension" was published in 2022. Journal: Int J Anal Chem.

### 3.6. Precision

In this study, both system and method precision such as repeatability and intermediate were evaluated. In case of system precision analysis, the RSD of retention time, peak area, and operating system of the chromatographic conditions revealed by the value of theoretical plates and tailing factors were observed to be lower than 2.0%. Furthermore, the number of theoretical plates was higher than 2000 for all analyte peaks, as given in Tables 6 and 7. Additionally, in case of method precision, the %RSD of assay value for CFX and CVA in assessment of repeatability and intermediate precision was obtained below 2.0%, which is given in Table 8. Thus, the data obtained for both system and method precision demonstrated that the method is precise, which is evidenced by the RSD and the tailing factor NMT 2.0%; similarly, the number of theoretical plates was NLT 2000.

### 3.7. Robustness

This testing parameter was analyzed by assessing the impact of slight alteration in chromatographic conditions. The data of robustness evaluation demonstrated that a minor modification of method conditions including flow rate and pH of mobile phase was found to be robust within the desired range (RSD less than 2.0%). The findings of CFX and CVA analysis are given in Tables 9 and 10. Furthermore, in all alterations, better separation of HPLC peak was observed between CFX and CVA. In addition, the RSD results of peak area achieved from repeated measurement of standard solution and percentage of assay for analytes received from sample solutions were found to be below 2.0%. At 1.2 mL/min of flow rate, the assay results for CFX and CVA were 99.65% and 100.43%, respectively. Moreover, there were no noticeable results observed when minor variations were applied in parameters (flow rate and pH).

### 3.8. Solution Stability

The recovery percentage was obtained within the acceptable limits of 98.0–102.0% and the %RSD was also NMT 2.0%. These results revealed that standard and sample solutions of both CFX and CVA were sufficiently stable for 24 h at two different conditions: 30°C and 4°C. Furthermore, the value of tailing factors and number of theoretical plates were found within acceptable range as well. The detailed results are given in Tables 11 and 12.

The article "A Validated RP-HPLC Method for Simultaneous Determination of Cefixime and Clavulanic Acid Powder in Pediatric Oral Suspension" was published in 2022. Journal: Int J Anal Chem.

## 4. Conclusion

In this research, a new, simple, accurate, precise, robust, and linear stability-indicating reverse phase HPLC method has been developed and validated for simultaneous assay evaluation of cefixime and clavulanic acid in pediatric oral powder formulation. Moreover, this analyzing method is validated as per the specification provided by ICH and proved to be appropriate for the intended application, able to give quantitative measurements accurately and precisely under slight variation of chromatographic conditions. This validated analytical method can support the pharmaceutical industries and other researchers to analyze cefixime and clavulanic acid containing dosage forms to evaluate quality in their products.

## Figures and Tables

**Figure 1:** Chromatogram of cefixime and clavulanic acid standard solution.

**Figure 2:** Chromatogram of cefixime and clavulanic acid sample solution.

**Figure 3:** Chromatogram of blank solution.

**Figure 4:** Chromatogram of placebo solution.

**Figure 5:** Calibration curve of cefixime.

**Figure 6:** Calibration curve of clavulanic acid.

**Table 1:** Results of method optimization.

Column	Mobile phase	Elution mode	Flow rate	pH	Observation	Result
C18	Methanol-water consists of disodium hydrogen phosphate (20 : 80, v/v)	Isocratic	1.0 mL/min	6.5	Poor resolution	Rejected
C18	Methanol-water consists of disodium hydrogen phosphate (20 : 80, v/v)	Isocratic	1.0 mL/min	6.0	Poor resolution	Rejected
C18	Methanol-water consists of disodium hydrogen phosphate (20 : 80, v/v)	Isocratic	1.0 mL/min	5.5	Good resolution	Accepted
C18	Methanol-water consists of disodium hydrogen phosphate (20 : 80, v/v)	Isocratic	1.0 mL/min	5.0	Poor and unstable peak shape	Rejected
C18	Methanol-water consists of disodium hydrogen phosphate (20 : 80, v/v)	Isocratic	1.0 mL/min	4.5	Poor and unstable peak shape	Rejected
C18	Methanol-water consists of disodium hydrogen phosphate (20 : 80, v/v)	Isocratic	1.0 mL/min	4.0	Poor and unstable peak shape	Rejected

**Table 2:** Specificity of cefixime.

S. no.	Retention time (minutes)		Area	
	Standard	Sample	Standard	Sample
1	7.268	7.110	1159.539	1171.232
2	7.245	7.099	1159.844	1170.727
3	7.226	7.089	1158.852	1172.009
4	7.208	7.079	1159.564	1172.305
5	7.190	7.070	1159.141	1172.559

Average	7.227	7.089	1159.388	1171.766
%RSD	0.420	0.224	0.0337	0.0653

**Table 3:** Specificity of clavulanic acid.

S. no.	Retention time (minutes)		Area	
	Standard	Sample	Standard	Sample
1	3.244	3.229	555.367	630.096
2	3.242	3.228	559.499	627.963
3	3.240	3.227	554.267	612.822
4	3.239	3.225	549.702	623.480
5	3.237	3.224	557.230	627.552

Average	3.240	3.227	555.213	624.383
%RSD	0.088	0.057	0.6601	1.1037

The article "A Validated RP-HPLC Method for Simultaneous Determination of Cefixime and Clavulanic Acid Powder in Pediatric Oral Suspension" was published in 2022. Journal: Int J Anal Chem.

**Table 4:** Accuracy analysis of cefixime.

% spiked level	Replicate number	Peak area	Assay (%)	Recovery (%)	Mean recovery (%)	SD	%RSD
80	1	918.459	78.69	98.36	98.30	0.06	0.061
	2	917.348	78.59	98.24			
	3	917.811	78.64	98.30			

100	1	1167.812	99.00	99.00	98.96	0.061	0.062
	2	1167.753	98.99	98.99			
	3	1166.553	98.89	98.89			

120	1	1418.013	121.68	101.40	101.54	0.132	0.130
	2	1420.387	121.88	101.57			
	3	1421.662	121.99	101.66			

**Table 5:** Accuracy analysis of clavulanic acid.

% spiked level	Replicate number	Peak area	Assay (%)	Recovery (%)	Mean recovery (%)	SD	%RSD
80	1	508.897	78.91	98.63	98.42	0.24	0.244
	2	508.080	78.78	98.48			
	3	506.474	78.53	98.16			

100	1	646.717	99.22	99.22	99.05	0.162	0.164
	2	645.420	99.02	99.02			
	3	644.587	98.90	98.90			

120	1	781.357	121.35	101.12	100.97	0.140	0.139
	2	779.162	121.00	100.84			
	3	780.143	121.16	100.96			

**Table 6:** System precision data from the cefixime standard solution of the proposed HPLC method.

Replicate number	RT	Peak area	Number of theoretical plates	Tailing factor
1	7.749	1139.443	2529.86501	1.03532
2	7.761	1152.379	2509.62483	1.03196
3	7.772	1152.066	2508.92684	1.03767
4	7.779	1150.464	2508.67867	1.03946
5	7.786	1150.183	2504.94281	1.04040
6	7.801	1149.996	2506.48037	1.04373

Average	7.775	1149.089	2511.42	1.038
%RSD	0.239	0.4203	—	—

**Table 7:** System precision data from the clavulanic acid standard solution of the proposed HPLC method.

Replicate number	RT	Peak area	Number of theoretical plates	Tailing factor	Resolution
1	3.287	570.210	4990.54925	1.40627	11.12753
2	3.288	569.841	4968.60734	1.38777	11.09475
3	3.289	569.613	4952.80516	1.40222	11.10328
4	3.289	568.535	4963.70704	1.40866	11.11486
5	3.290	568.181	4958.28079	1.40111	11.11313
6	3.291	567.685	4956.35583	1.41483	11.13316

Average	7.775	1149.089	4965.051	1.403	11.114
%RSD	0.239	0.4203	—	—	—

**Table 8:** Results of repeatability and intermediate precision.

No. of sample solutions	Sample weight (g)	Content of cefixime in oral powder (%, compared to labeled claim)	Content of clavulanic acid in oral powder (%, compared to labeled claim)
Day 1, analyst 1			
1	5.5100	99.00	100.43
2	5.5012	99.01	100.16
3	5.5006	99.11	100.33
4	5.5123	98.88	99.68
5	5.5198	98.82	99.61
6	5.5118	98.98	98.92
Average (1–6)		98.97	100.02
%RSD (1–6)		0.1051	0.3402

Day 2, analyst 1			
7	5.5100	98.60	99.85
8	5.5012	99.40	99.41
9	5.5006	98.39	99.47
10	5.5123	99.82	99.48
11	5.5198	99.35	99.15
12	5.5118	98.94	98.44
Average (7–12)		99.08	99.47

%RSD (7–12)		0.5437	0.2232

Day 2, analyst 2			
13	5.5088	98.71	100.15
14	5.5069	99.08	99.48
15	5.5006	98.83	99.41
16	5.5108	99.37	99.52
17	5.5029	99.48	99.39
18	5.5105	98.04	99.21
Average (13–18)		98.92	99.53
%RSD (13–18)		0.3806	0.3259

The article "A Validated RP-HPLC Method for Simultaneous Determination of Cefixime and Clavulanic Acid Powder in Pediatric Oral Suspension" was published in 2022. Journal: Int J Anal Chem.

**Table 9:** Robustness data of the proposed HPLC method for cefixime.

Parameters		Avg. std. area (*n* = 6)	%RSD of std. area	Avg. sample area (*n* = 6)	%RSD of sample area	%assay (*n* = 6)	%RSD of assay
Flow rate	0.8 mL/min	1446.738	0.0370	1179.034	0.2931	101.07	0.4145
	1.2 mL/min	958.232	0.1247	971.292	0.2592	99.65	0.3118

pH	5.3	1149.024	0.0992	1155.507	0.0380	98.86	0.1525
	5.7	1152.101	0.0962	1168.877	0.2503	99.74	0.2454

**Table 10:** Robustness data of the proposed HPLC method for clavulanic acid.

Parameters		Avg. std. area (*n* = 6)	%RSD of std. area	Avg. sample area (*n* = 6)	%RSD of sample area	%assay (*n* = 6)	%RSD of assay
Flow rate	0.8 mL/min	690.375	0.0970	777.192	0.4834	99.74	0.5246
	1.2 mL/min	458.453	0.7325	519.788	0.6229	100.43	0.4519

pH	5.3	548.329	0.2196	620.548	0.1804	100.27	0.2610
	5.7	541.271	0.1995	610.756	0.3764	99.98	0.4910

**Table 11:** Solutions stability data of the proposed HPLC method for cefixime.

Parameter	Stability conditions	RT	Avg. peak area	%RSD (peak area)	Tailing factor	Assay (%)	%RSD (assay)	Number of theoretical plates
Standard solution	0 h	7.68	1102.022	0.1573	1.065	—	—	2566.332
	After 24 h at 30°C	7.19	1103.382	0.0854	1.134	—	—	2553.285
	After 24 h at the refrigerator	7.30	1159.015	0.0246	1.10	—	—	2556.207

Sample solution	0 h	7.52	1108.138	0.3846	1.11	98.85	0.3721	2382.315
	After 24 h at 30°C	7.37	1108.723	0.0506	1.16	98.74	0.1475	2370.762
	After 24 h at the refrigerator	7.43	1167.680	0.0506	1.10	99.04	0.1610	2438.755

**Table 12:** Solutions stability data of the proposed HPLC method for clavulanic acid.

Parameter	Stability conditions	RT	Avg. peak area	%RSD (peak area)	Tailing factor	Assay (%)	%RSD (assay)	Number of theoretical plates
Standard solution	0 h	3.28	531.098	0.9661	1.459	—	—	5065.394
	After 24 h at 30°C	3.24	517.890	0.3458	1.504	—	—	4948.156
	After 24 h at the refrigerator	3.24	558.564	0.5773	1.516	—	—	4868.868

Sample solution	0 h	3.27	596.532	0.3130	1.467	99.52	0.4378	5080.242
	After 24 h at 30°C	3.25	580.709	0.2932	1.511	99.35	0.3840	4918.414
	After 24 h at the refrigerator	3.25	635.529	0.4743	1.504	100.81	0.5608	4806.592

## Data Availability

No external data were used to support this study.
